# Epileptic Seizure Detection with Hybrid Time-Frequency EEG Input: A Deep Learning Approach

**DOI:** 10.1155/2022/8724536

**Published:** 2022-02-15

**Authors:** Yayan Pan, Xiaoyu Zhou, Fanying Dong, Jianxiang Wu, Yongan Xu, Shilian Zheng

**Affiliations:** ^1^Department of Emergency Medicine, The Second Hospital of Jiaxing, Jiaxing 314000, China; ^2^Department of Emergency Medicine, The Second Affiliated Hospital Zhejiang University School of Medicine, Hangzhou 310009, China; ^3^State Key Laboratory of Integrated Service Networks, Xidian University, Xi'an 710071, China; ^4^No. 011 Research Center, Science and Technology on Communication Information Security Control Laboratory, Jiaxing 314033, China

## Abstract

The precise detection of epileptic seizure helps to prevent the serious consequences of seizures. As the electroencephalogram (EEG) reflects the brain activity of patients effectively, it has been widely used in epileptic seizure detection in the past decades. Recently, deep learning-based detection methods which automatically learn features from the EEG signals have attracted much attention. However, with deep learning-based detection methods, different input formats of EEG signals will lead to different detection performances. In this paper, we propose a deep learning-based epileptic seizure detection method with hybrid input formats of EEG signals, i.e., original EEG, Fourier transform of EEG, short-time Fourier transform of EEG, and wavelet transform of EEG. Convolutional neural networks (CNNs) are designed for extracting latent features from these inputs. A feature fusion mechanism is applied to integrate the learned features to generate a more stable syncretic feature for seizure detection. The experimental results show that our proposed hybrid method is effective to improve the seizure detection performance in few-shot scenarios.

## 1. Introduction

Approximately one percent of the world's population, 65 million people, suffer from epilepsy, more than Parkinson's disease, Alzheimer's disease, and multiple sclerosis combined [1]. About two-thirds of people with epilepsy can be treated with medication, and the rest may require surgical intervention. Epilepsy has the characteristics of sudden and recurrent seizures, which may lead to falls, asphyxia, and even death. Therefore, seizure detection is very important for early warning and treatment of epilepsy.

Epileptic seizure detection is mainly based on electroencephalogram (EEG) [2–4]. Single-channel EEG acquisition equipment improves the practicability of EEG in epileptic detection due to its simplicity in implementation. However, the provided information by signal-channel EEG signal is limited because of the small number of channels. Therefore, it is worth studying to establish a model with high accuracy and high robustness for single-channel EEG epileptic detection.

The traditional methods are mainly based on feature engineering techniques which extract the corresponding features from EEG signals and then complete the detection based on the extracted features [5–9]. These features include time-domain features [10–12], frequency-domain features [8, 9], and time-frequency-domain features [13–15]. Once the features are extracted, EEG signals can be classified using a variety of classifiers. No matter what classifier is used, the quality of designed features will greatly affect the performance of epilepsy detection. In recent years, with the development of deep learning technology, many works have applied deep learning to perform epilepsy detection [16, 17]. Different from traditional feature engineering, deep learning methods automatically learn features from EEG signals and further complete detection tasks with an end-to-end manner without complicated manual feature design process and can achieve better performance than traditional methods in many scenarios.

The EEG signal input forms used by these deep learning methods are varied, including time-domain input, frequency-domain input, and time-frequency-domain input (including short-time Fourier transform (STFT) and wavelet transform).

Specifically, as for time-domain input, in [18], the authors applied convolutional neural network (CNN) to design an autoencoding framework in order to learn unsupervised features from EEG signals. This unsupervised learning method automatically transforms the time-domain EEG sequences into low-dimensional features which facilitates the classification of EEG signals. Long short-term memory (LSTM) network was used in [19] for seizure detection without transforming the EEG data into other forms. It directly discovered discriminative temporal patterns from the raw EEG data.

In addition to the time series, the input format in frequency domain has also been explored. The frequency spectrogram obtained by fast Fourier transform (FFT) was treated as the input of CNN for the purpose of epileptic detection in [20]. The subband mean amplitude of spectrum map (MAS) obtained from different EEG rhythms was adopted for EEG representation in [21], and stacked CNNs were used for feature extraction and seizure detection. It proved that the MAS has the ability to characterize the different rhythms of EEG signals.

Recently, it has appeared growing interest in using time-frequency image to implement seizure detection since the time-frequency image can provide more detailed contextual information compared with the time-domain input. In [22], the authors adopted STFT to transform the segmented EEG signals into 2-D spectrogram fragments and designed a deep learning framework to extract latent features for performing seizure detection. It showed that the performance using time-frequency image is better than that using time-domain input because the clear energy distribution in the time-frequency distribution helps the classifier to capture more useful information.

Wavelet transform can also be used to obtain the time-frequency properties. Different from the fixed length of window function used in STFT, the wavelet transform uses short-time window at high frequency while using long-time window at low frequency, which is helpful to obtain good localization characteristics in both time domain and frequency domain. In [23], the authors used CNN to learn quantitative signatures from the wavelet transform of EEG signals for distinguishing the preictal, ictal, and interictal states.

Although deep learning can automatically learn features from the input signals, however, different input formats will still affect the final epilepsy detection performance. For example, it has been pointed out in [20, 22] that the detection performance of time-domain input is worse than that of frequency-domain input. In [24], the authors focused on deep multiview feature extraction from Fourier transform and wavelet packet decomposition of EEG signal as well as the time-domain signal for seizure detection. However, from these works, we are not sure which EEG input format is the best for deep learning-based seizure classification. To solve this problem, a hybrid method is proposed in this paper. We explore to take various formats of EEG signals as input and hand them to a deep neural network for feature extraction, which will help to classify epilepsy. Different from the method in [24], which firstly trained independent neural networks to construct deep multiview feature from the initial multiview features and then learned a multiview classifier for recognizing the EGG signal based on the aforementioned deep multiview feature, our proposed network jointly optimize subnetworks used for processing different domain inputs and the whole network can be regarded as a classifier; it thereby does not require to train an additional classifier anymore. On the other hand, the process of joint training allows the network to adaptively adjust each subnetwork for learning corresponding dependence among subnetworks. In addition, most prior works assumed there are adequate samples for training. However, the labeled EEG samples with seizures are difficult to acquire in real-life. Different from prior works, we will consider few-shot scenarios in this paper where there are only a small number of samples available for training the deep learning model for epilepsy detection. A large number of experiments are conducted to verify the performance of the proposed method. Specifically, the main contributions of this paper are as follows:

- We propose an epilepsy detection method based on deep learning with hybrid input formats of EEG signals, i.e., original EEG, DFT, STFT, and DWT of EEG. In the proposed framework, we use four individual CNNs to extract features from the multiple-domain input. A feature fusion mechanism is adopted to integrate the learned features to generate a syncretic feature, which is considered to be more stable and superior for epilepsy classification than the features extracted from single-domain input
- We focus on epilepsy diagnosis using the deep learning method in few-shot scenario where adequate epileptic ictal EEG is not available. To alleviate the tendency of overfitting to the data, we design lightweight CNNs which are based on depthwise separable convolution and add a regularization term for decreasing the complexity of the deep learning model
- We conduct experiments to verify the performance of our proposed method. Benefited from the complementarity of the properties of EEG signal in time domain and frequency domain, our proposed method achieves higher-accuracy performance of epilepsy classification compared with the methods using single input

## 2. Materials and Methods

In this section, firstly, we briefly introduce the four representations of EEG signal in time domain, frequency domain, and time-frequency domain: raw EEG signal, Fourier transform, short-time Fourier transform, and wavelet transform of EEG signal. Then, we describe our proposed deep learning model based on lightweight network for epilepsy classification.

### 2.1. Raw EEG Signal

As discussed before, EEG is an effective technology for epilepsy diagnosis. EEG can reveal complex brain functions, such as cognition, emotion, attention, and memory through capturing voltage changes generated by neuronal activity in the brain. In reality, the EEG signals collected by EEG equipment need to be processed by analog-to-digital converters, so the EEG signals are sampled at discrete time points, which can be represented as

(1) $$\begin{array}{c} x\left(n\right)=x\left(t\right)\delta_{T}\left(t\right), \end{array}$$

where *x*(*t*) is the EEG signal in analog domain, *δ*_*T*_(*t*) is the impulse function, *T* = 1/*F*_*s*_ is the sampling period, and *F*_*s*_ is the sampling frequency. The EEG signals may be disturbed by other physiological signals and spatial electromagnetic noise. The information contained in EEG signals is complicated. Therefore, we try to analyze it from a different perspective other than single time domain, for instance, in frequency domain or time-frequency domain as discussed in the following.

### 2.2. Fourier Transform of EEG Signal

Fourier transform has been widely adopted for analyzing the spectrum of various signals in the field of signal processing. As the EEG signal contains complex frequency information during seizures, it is feasible to perform Fourier transform on EEG signals for obtaining information in frequency domain. For a discrete EEG signal *x*(*n*), the definition of discrete Fourier transform (DFT) [25] is

(2) $$\begin{array}{c} X\left(k\right)=\overset{N-1}{\underset{n=0}{\sum }}x\left(n\right)e^{-j2\pi kn/N},\;k=0,1,\cdots ,N-1, \end{array}$$

where *N* represents the sampling points of EEG signal and *X*(*k*) is the obtained sequence in frequency domain after DFT. The Fourier transform has its limitation on processing nonstationary signal, whose frequency is varying with time. The Fourier transform can only tell the contained frequency components of the signal; however, the corresponding frequency at each time moment is not available. Time-frequency transform is needed to obtain such information.

### 2.3. Short-Time Fourier Transform of EEG Signal

In spectrum analysis, we assume that the spectrum of the EEG signal is not varying with time. Apparently, this assumption simplifies the nonstationary and dynamic characteristics of EEG signals. In fact, the EEG signals are highly nonstationary, which means that the statistical properties and spectral density of EEG signals change over time. The STFT can be sued for analyzing nonstationary signal and transform the time sequence into time-frequency domain. The main idea of STFT is regarding a nonstationary signal as a stack of several truncated short-time stationary signals. This process is achieved by windowing the original signal and segmenting the signal into several fixed-length signals in time domain. For each truncated signal, it can be approximately regarded as a stationary signal, and thus, Fourier transform can then be used. The discrete STFT [21] can be expressed by

(3) $$\begin{array}{c} X_{n}\left(k\right)=\overset{+\infty }{\underset{m=-\infty }{\sum }}x\left(m\right)w\left(n-m\right)e^{-j2\pi km/N},\;k=0,1,\cdots ,N-1, \end{array}$$

where *w*(*n* − *m*) is the window function. The result of STFT is a 2-D spectrogram. In general, the latent features in the time-frequency domain of EEG signals are easier to be learned for deep learning than the features of EEG signals in time domain.

### 2.4. Wavelet Transform of EEG Signal

The fixed-length window in STFT will induce the fixed time-frequency resolution and cannot adapt to diversified signal components. In general, the EEG signal is composed of short-duration high-frequency components and long-duration low-frequency components. Therefore, the time-frequency analysis of EEG signal requires a more adaptive time-frequency resolution. The wavelet transform is a popular time-frequency analysis method, which adopts an optimized strategy of window choosing: using short-time window at high frequency while using long-time window at low frequency. An important property of wavelet transform is that it has good localization characteristics in both time domain and frequency domain. The wavelet transform obtains the time information of the signal by shifting the mother wavelet and obtains the frequency characteristics of the signal by scaling the wavelet. For the discrete wavelet transform (DWT), given a discrete signal *x*(*n*) with length *N*, a pair of wavelet decomposition filters related to a specific mother wavelet is used to perform wavelet analysis. The one-level DWT [26] is expressed by the following equations:

(4) $$\begin{array}{c} {cA}_{1}=X_{LoD}*x\left(n\right)\delta \left(t-2n\right), \end{array}$$

(5) $$\begin{array}{c} {cD}_{1}=X_{HiD}*x\left(n\right)\delta \left(t-2n\right), \end{array}$$

where *cA*_1_ is the approximation coefficients of one-level DWT, *cD*_1_ is the returned detail coefficients, *X*_*LoD*_ is the lowpass filter, *X*_*HiD*_ is the high-pass filter, ∗ represents the convolution operation, and *δ*(*t* − 2*n*) is the pulse function, and it means the results of a filter are downsampled with factor 2. For multilevel DWT, the coefficients *cA*_*j*_ and *cD*_*j*_ are produced through replacing the input *x*(*n*) by *cA*_*j*−1_. In general, the compositions of DWT analyzed at level *j* contain the following coefficients: [*cA*_*j*_, *cD*_*j*_, ⋯, *cD*_1_].

## 3. Proposed Epilepsy Classification Method

Different from the aforementioned methods that only use a single representation of the EEG signal, we are interested in combining the information in time domain with information in frequency domain to benefit from the complementarity of both. Meanwhile, considering the general deep learning models in few-shot scenario will induce the undesirable tendency to extremely overfit the data, we try to build our model based on lightweight network to alleviate this tendency.

### 3.1. Designed Deep Learning Framework for Epilepsy Classification

The block diagram relationship of our designed deep learning model is shown in Figure 1, which can be decomposed into four parts, namely, hybrid input acquisition, feature extraction, feature fusion, and softmax output. The details of our proposed algorithm will be introduced in these four parts.

#### 3.1.1. Hybrid Input Acquisition

In this part, the raw EEG signal was used to calculate the hybrid input format, containing the aforementioned DFT, STFT, and DWT of EEG. In general, signal-domain representation of signal is too limited to distinguish different signals. The main purpose of this part is to transform the time-domain EEG signal to frequency-domain and time-frequency-domain representation, obtaining a rich representative format of EEG signal in different domains. Equations (2)–(5) show the mathematical calculation of hybrid input.

#### 3.1.2. Feature Extraction

Feature extraction is a critical part of the DL-based detection algorithm as the quality of extracted feature will determine the performance of detection. In this paper, CNN is chosen as a feasible scheme for extracting features from the hybrid inputs for two reasons. On the one hand, the scale structure and regional interaction characteristics of CNN are relatively consistent with signals with local characteristics, time-varying character of EEG signal for example. On the other hand, after STFT, the generated two-dimensional spectrogram can be regarded as image actually, motivated by the superior performance of CNN in the field of image recognition; it is proper to adopt CNN to learn the adjacent relation in the two-dimensional image.

In this paper, we provide a feasible framework for feature extraction, as shown in Figure 2, where four individual CNNs are used to extract features from their own corresponding input. After several layers of lightweight CNN, feature maps corresponding to each input are generated, followed by global average pooling layers, whose function is transforming the feature maps into feature vectors. It should be noted that the adopted feature extractor can be replaced by other superior neural networks, depending on the selected hybrid input.

#### 3.1.3. Feature Fusion

The aim of feature fusion is to generate more discriminate feature representation from several individual feature vectors. In Figure 2, the feature vectors originated from four different inputs are integrated together to produce a syncretic feature vector. This process is called feature fusion, which vertically appends the features and can be represented as

(6) $$\begin{array}{c} F=F_{1}⊕F_{2}⊕F_{3}⊕F_{4}, \end{array}$$

where *F* is the syncretic feature, *F*_1_, *F*_2_, *F*_3_, and *F*_4_ are feature vectors corresponding to the four inputs, and ⊕ is the connection function, which stacks the corresponding features. The syncretic feature vector is considered to be more stable than a single feature vector because this structure can make full use of the advantages of each input information. Furthermore, when some of the feature vectors among *F*_1_, *F*_2_, *F*_3_, and *F*_4_ performs wore than the rest, then, their allocated weights will have the tendency to be smaller for avoiding bringing too much damage to the final performance.

#### 3.1.4. Softmax Output

The decision about epilepsy seizure is modeled as a binary classification problem where label “0” represents the result is normal and label “1” represents the result is epileptic. A fully connected layer with two neurons which are normalized by softmax activation function is then served as giving the probabilities belonging to each category:

(7) $$\begin{array}{c} {\hat{p}}_{i}=\frac{e^{x_{i}}}{\sum_{j=1}^{2}e^{x_{j}}},\;i=0,1, \end{array}$$

where ${\hat{p}}_{i}$ is the normalized probability belonging to category *i*. In the binary classification problem, when ${\hat{p}}_{0}>{\hat{p}}_{1}$, it means that the predicted result is normal; otherwise, the predicted result is epileptic.

In order to alleviate the tendency of overfitting to the data, *l*2 regularization is applied, whose function is decreasing the complexity of the model. The regularization term is actually treated as a penalty, and it is used to limit the parameters specified by loss function for preventing large values of the parameters. When *l*2 regularization is added, the model with simultaneous low prediction loss and low complexity will be chosen as the optimal model, and it can be represented as

(8) $$\begin{array}{c} w^{*}=\arg\underset{w}{\min}\overset{c}{\underset{i=1}{\sum }}p\left(x_{i}\right)\log\left(q\left(x_{i}\right)\right)+\lambda \overset{k}{\underset{i=1}{\sum }}w_{i}^{2}, \end{array}$$

where *λ* defines the degree of penalty, which is set to be 10^−4^ in this paper, **w**^∗^ is the chosen optimal parameters in the deep learning model, ∑_*i*=1_^*c*^*p*(*x*_*i*_)log(*q*(*x*_*i*_)) is the commonly used cross-entropy loss for classification problem, *p*(*x*_*i*_) represents the true probability belonging to the *i*th class, *q*(*x*_*i*_) represents the predicted probability belonging to the *i*th class, and *c* is the number of classes which is equal to 2 for epilepsy classification problem in this paper.

### 3.2. Lightweight CNN

Recently, lots of superior CNN structures have been proposed, such as ResNet and DenseNet. These models have achieved remarkable performance in image classification, which is benefited from the models' strong ability to supervise learning. However, these deep learning models require a large number of labeled samples to construct an effective classification model. When the labeled samples are insufficient, which is known as few-shot scenario, these models will suffer from severe performance loss. The imbalance between large number of parameters of the model and few labeled training samples is the crucial problem to be handled for few-shot classification. In our designed deep learning framework, we adopt lightweight convolution to replace the traditional convolution for reducing the parameters of the model. The lightweight convolution is often referred to as depthwise separable convolution, which is a combination of depthwise convolution and pointwise convolution. In the process of depthwise convolution, the number of kernels is identical to the number of the channels of input, and each kernel is convoluted with its feature map (one channel is regarded as one feature map). The depthwise convolution is a special situation of group convolution where each channel of input is regarded as one group.  Figure 3 shows the depthwise convolution with 3 groups. We can see that the relation among feature maps is neglected and the convolutions in groups are independent during depthwise convolution. For remedying this shortcoming, the second stage of depthwise separable convolution, pointwise convolution, uses the traditional convolution to ensure the interchange among feature maps. For reducing the parameters of convolution, it usually uses a convolution kernel with a size of 1 × 1. The depthwise separable convolution can be expressed as

(9) $$\begin{array}{c} D_{i}=I_{i}⊗G_{i}, \end{array}$$

(10) $$\begin{array}{c} P_{m}=\underset{i}{\sum }D_{i}⊗K_{m,i}, \end{array}$$

where *D*_*i*_ ∈ ℝ^*m*×*n*^ represents the *i*th depthwise features after depthwise convolution, *I*_*i*_ is the *i*th channel of input, *G*_*i*_ is the convolution kernel of the *i*th group in depthwise convolution, ⊗ denotes the operation of convolution, *K*_*m*,*i*_ represents the kernel with a size of 1 × 1, and *P*_*m*_ is the *m*th pointwise features after pointwise convolution.

As the EEG signal is 1-D time sequence while the result of STFT is 2-D time-frequency image, two different structures of CNNs for feature extraction are built, which are shown in Figure 4. “Conv, 16, 31 × 1” indicates this convolution layer is the traditional convolution with 16 kernels and the kernel size is 31 × 1 while “DConv” represents the depthwise separable convolution. Note that the “Conv” layer shown in the figure corresponds to the sequence Conv-BN- (batch normalization-) ReLu. “Max_pool” denotes the maximum pooling layer with stride 2, and “Global_Avg pool” is the global average pooling layer which has no parameter to optimize. We can see that the most obvious distinction between the two structures for feature extraction from Figures 4(a) and 4(b) is the kernel size used in each convolution layer. For 1-D input, the kernel size is shaped as *N* × 1 while for 2-D input, the kernel size is shaped as *N* × *M* (*M* ≠ 1).

## 4. Results and Discussion

We focus on epilepsy classification using multiple time-domain and frequency-domain information in order to improve the performance of seizure detection. In this section, we first discuss the used EEG dataset, and then, we discuss the performance of our proposed method in few-shot scenario.

### 4.1. Dataset and Parameter Settings

In this paper, the adopted dataset is acquired online, which is published by Andrzejak et al. [27]. The dataset is composed of five categories, expressed by A, B, C, D, and E. Each category contains 100 recorded EEG signals using a standard 10-20 electrode placement system. The length of each EEG signal is 4097. The samples in category A and category B are collected from five healthy volunteers, and the discrimination between the two categories depends on whether the volunteer is eye opened (A) or eye closed (B). Category C and category D contain the interictal epileptic signals, which are measured on five epilepsy patients. The samples in category C are taken from the hippocampal formation of the opposite hemisphere of the brain while the samples in category D are taken from the epileptogenic zone. Category E records epileptic ictal EEG in the intracranial epileptogenic zone.

In the process of STFT, Hamming window is used to divide the signal into segments, and the length of window is set to be 128. It uses 128 sampling points to calculate the discrete Fourier transform and 120 sampling points for its overlap between adjoining segments. Besides, we perform two-level DWT on EEG signal using the “db1” wavelet, whose results have the following structure: [*cA*_2_, *cD*_2_, *cA*_1_]. We choose one sample from category A and category E, respectively, as an example to show the results of the four representations of EEG signals. Figures 5(a) and 5(b) show the normal EEG signal (A) and epileptic ictal EEG signal (E), respectively. The normal EEG signal is a transient waveform, and it has distinct peaks. Figures 5(c)–5(h) illustrate the amplitude of the FFT, STFT, and DWT of the EEG signals. Comparing Figures 5(c) and 5(d), we can see that the maximum amplitude of spectrum appears in *θ* rhythm for normal EEG and in *δ* rhythm for epileptic ictal EEG. The peak value corresponding to epileptic ictal EEG is much bigger than the normal EEG's. As for the results of STFT, it can be seen from Figures 5(e) and 5(f) that the power in *δ*, *α*, and *β* rhythm of epileptic ictal EEG is obviously larger than that of normal EEG. The results of DWT are concatenated together as the input of CNN, which are shown in Figures 5(g) and 5(h).

### 4.2. Configuration Details

In this paper, our proposed neural network has four branch networks, which are used to process and extract features from inputs of different domains, deleting or adding branch network to adapt to the variety of inputs according to the number of input types. Each branch network contains five convolution layers, every one of which is followed by BN layer and ReLu layer. The momentum in each BN layer is set to 0.9. It is not wise to use too many kernels in our proposed network, which will result in a highly parameterized network and overfitting problem. It can be seen that we only use 16 and 32 kernels in each layer for alleviating overfitting. Except that the first convolution uses a large receptive field (31 × 1, 15 × 7) in order to obtain a long-distance relationship, the receptive field in the rest of convolution is 3 × 1. In each branch network, after the operation of global average pooling, it will generate a 32-dimensional feature vector corresponding with input of each domain. As a result, the concatenate of four feature vectors generate a 128-dimensional feature vector for the final decision. Furthermore, our experiments are conducted with Keras 2.3.1 and the neural network is trained on NVIDIA GeForce RTX 2080. During training, the batch size is set 6 and the maximum number of epochs is set 100. The initial learning rate is 0.005, and after every 20 epochs, the learning rate drops to 1/2 of the previous learning rate. Adam optimizer is adopted for optimizing the loss function.

### 4.3. Results

For validating the effectiveness of our proposed method, we compare the classification performance of the proposed method with four methods using single input, EEG, FFT, STFT, and DWT, respectively. In this paper, we focus on binary classification problem for distinguishing the normal EEG signals and epileptic EEG signals. Cross-validation is performed on the dataset for ensuring the reliability of validation. For fair comparison, two metrics are adopted to measure the performance in different scenarios, average accuracy, and variance. Average accuracy is calculated by averaging the results of *N*-fold cross-validation. Variance is adopted to reflect the stability of classification for *N*-fold cross-validation. We know that the large fluctuation of classification accuracy of *N*-fold cross-validation will induce large variance.

We first verify the performance of classifying normal and seizure EEGs (A vs. E).  Table 1 shows the results of different methods with 5-fold cross-validation, in which a total of 40 samples (20 samples for each category) are used for training and 160 samples for validation. It can be seen from the simulation results that among the four methods with single input, the classification accuracy of DWT input and STFT input is close and is higher than that of original EEG input, while the accuracy of FFT input is the lowest. Among the four scenarios with single input, the variance of DWT is the smallest, which means that the fluctuation of diagnosis accuracy of 5-fold cross-validation is the smallest and the performance of the method with DWT input is the most stable. From the performance comparison of the four methods with single input, we can conclude that the time-frequency-domain information is more discriminative for seizure detection compared with the frequency-domain information and time-domain information. When hybrid input is considered, the classification accuracy is further improved to 0.9912, which has almost 1% improvement in diagnosis accuracy compared with the method with the DWT method, and the variance is further decreased to 0.0034. The obtained simulation results in Table 1 validate the superiority of our proposed method.

In order to evaluate the effect of the number of training samples on the classification accuracy, we train the network with 10-fold cross-validation (the total number of training samples is 20) and 20-fold cross-validation (the total number of training samples is 10), respectively. The validation results are shown in Tables 2 and 3. Similarly, we can see that the performance of the method with single DWT input and single STFT input is still better than that of the method with single time-domain EEG input, and the proposed method with hybrid input obtains the best classification accuracy and the smallest variance. From another perspective, when the number of training samples decreases from 40 to 20, the classification accuracy of the method with single EEG input has 2% performance loss, decreased from 0.9738 to 0.9534, while the performance loss for the proposed method with hybrid input is 1.2%, decreased from 0.9912 to 0.9794. Furthermore, when the number of training sample decreases to 10, it only has slight performance loss for the method with EEG input and the method with DWT input; however, the performance of the method with STFT input has a huge decrease. Overall, our proposed method performs the best in terms of average classification accuracy and variance in the two experiments (10-fold cross-validation and 20-fold cross-validation) which further validates the superiority of our proposed method.

In order to further verify the effectiveness of the hybrid input for the epilepsy detection, we compare the performance of signal-domain input with that of hybrid input. In addition to the feature extractor that we designed in this paper, we have also considered another feature extractor proposed in [28], where LSTM was used to extract seizure-associated features. We consider the combination of raw EEG data, DFT sequence, and the DWT sequence as the hybrid input when the LSTM is adopted. The accuracy in Table 4 is obtained through 20-fold cross-validation. According to the performance comparison, we can see that the LSTM obtains better detection performance compared with the CNN, which illustrates that the LSTM is more suitable for processing the temporal sequence. Furthermore, when the hybrid input was used as the input of LSTM, the detection performance can be further improved, which proves that the hybrid input is helpful to improve the performance of epilepsy detection. Moreover, we give the detection time for each signal, which has 23.6-second duration. From the simulation results, we can see that the detection time is much smaller than the duration of the EEG signal.

In the last experiment, we verify the performance of the proposed method in distinguishing the normal and nonseizure (AB vs. CD) with 10-fold cross-validation.  Table 5 provides the results. Similarly, in Table 5, the first four rows give out the diagnosis accuracy of 10-fold cross-validation, the average diagnosis accuracy, and the variance of diagnosis accuracy of 10-fold cross-validation for four methods with single input. It can be seen from the obtained experimental data of the first four rows in Table 5, different from the case of A vs. E, where among the three methods with single input, the DWT and STFT achieve higher classification accuracy than the EEG input; the EEG input gets the highest classification accuracy in the case of AB vs. CD. Once combining the four input formats as the hybrid input of our proposed network, the diagnosis accuracy is obviously improved, about 0.86% increase in average diagnosis accuracy compared with that of the method using time-domain input solely, about 16% increase in average diagnosis accuracy compared with that of the method using frequency-domain input solely. Furthermore, the method with hybrid input gets the smallest variance among the five methods, which means that the fluctuation of diagnosis accuracy of 10-fold cross-validation is the smallest and therefore demonstrates the performance of our proposed method is stable. Thus, simulation results can demonstrate that our proposed method with hybrid input has strong advantages whether in average accuracy or variance, which proves the effectiveness of the proposed method in epileptic classification.

## 5. Conclusions

In this paper, we focus on epileptic classification in few-shot scenarios. In order to make the classification accuracy higher and more stable, we propose a deep learning method with hybrid input, i.e., original EEG signal, FFT, STFT, and DWT of EEG signal. In order to alleviate the tendency of overfitting, two means are applied. The first is that we replace the traditional convolution by depthwise separable convolution for reducing the parameters in network and then *l*2 regularization is applied, whose function is decreasing the complexity of the model. We conduct several experiments to distinguish normal and epileptic EEG, and the results show the proposed method with hybrid input has strong advantages in epileptic classification. It benefits from the complementarity of time-domain properties, frequency-domain properties, and time-frequency-domain properties. Our proposed method provides a new perspective to enrich the input information to make improvements for deep learning-based epileptic diagnosis.

## Figures and Tables

**Figure 1:** The block diagram of the proposed method for epilepsy classification.

**Figure 2:** The designed deep learning framework for epilepsy classification.

**Figure 3:** The process of depthwise separable convolution.

**Figure 4:** Structures of CNNs for feature extraction: (a) CNN with 1-D input and (b) CNN with 2-D input.

**Figure 5:** The EEG signal and the amplitude of complex-valued STFT and DWT of the EEG signal: (e) STFT of A, (f) STFT of E, (g) DWT of A, and (h) DWT of E.

**Table 1:** Performance of normal vs. seizure case (A vs. E) with 5-fold cross-validation.

Methods	K1	K2	K3	K4	K5	Mean	Variance
EEG	0.9563	0.9563	0.9688	0.9937	0.9937	0.9738	0.0189
DWT	0.96875	0.9875	1.0	0.9812	0.9750	0.9825	0.0120
FFT	0.9312	0.9312	0.8438	0.9812	0.9500	0.9275	0.0510
STFT	0.9875	1.0	0.95	0.9875	1.0	0.9850	0.0205
Hybrid	0.9875	0.9937	0.9937	0.9937	0.9875	0.9912	0.0034

**Table 2:** Performance of normal vs. seizure case (A vs. E) with 10-fold cross-validation.

Methods	K1	K2	K3	K4	K5	K6	K7	K8	K9	K10	Mean	Variance
EEG	0.9556	0.9667	0.9778	0.9278	0.9611	0.9167	0.9667	0.9556	0.9444	0.9611	0.9534	0.0187
DWT	0.9278	0.9389	0.9833	0.9611	0.9889	0.9833	0.9667	0.9833	0.9444	0.9667	0.9644	0.0213
FFT	0.9222	0.9889	0.9889	0.9722	0.9667	1.0	0.9833	0.8944	0.8556	0.9944	0.9567	0.0491
STFT	0.9222	0.9778	0.95	0.9222	1.0	0.9889	0.9389	1.0	0.9778	0.9667	0.9644	0.0297
Hybrid	0.9667	0.9667	0.9944	0.9722	0.9778	0.9611	0.9833	0.9944	0.9944	0.9833	0.9794	0.0125

**Table 3:** Performance of normal vs. seizure case (A vs. E) with 20-fold cross-validation.

Methods	K1	K2	K3	K4	K5	K6	K7	K8	K9	K10	K11	K12
EEG	0.9556	0.9667	0.9778	0.9278	0.9611	0.9167	0.9667	0.9556	0.9444	0.9611	0.9536	0.9737
DWT	0.9278	0.9389	0.9833	0.9611	0.9889	0.9833	0.9667	0.9833	0.9444	0.9667	0.9579	0.9579
FFT	0.9222	0.9889	0.9889	0.9722	0.9667	1.0	0.9833	0.8944	0.8556	0.9944	0.9895	0.9895
STFT	0.9222	0.9778	0.95	0.9222	1.0	0.9889	0.9389	1.0	0.9778	0.9667	0.9158	0.9789
Hybrid	0.9667	0.9667	0.9944	0.9722	0.9778	0.9611	0.9833	0.9944	0.9944	0.9833	0.9579	0.9579
Methods	K13	K14	K15	K16	K17	K18	K19	K20	Mean	Variance		
EEG	0.9737	0.9684	0.9474	0.9947	0.8842	0.9684	0.9474	0.9895	0.9498	0.0297		
DWT	0.9947	0.9368	0.9895	0.9579	0.9474	0.9947	0.9579	0.9895	0.9595	0.0292		
FFT	0.9895	0.9947	0.9947	0.9789	0.9947	1.0	0.9947	0.9842	0.9371	0.12		
STFT	0.8368	0.7895	0.9632	1.0	0.9053	0.8947	0.9947	0.9684	0.9431	0.0564		
Hybrid	0.9895	0.9789	0.9526	0.9947	0.9421	0.9736	0.9684	0.9789	0.9639	0.0267		

**Table 4:** Performance of hybrid input using LSTM.

Methods	EEG	DWT	FFT	STFT	Hybrid	EEG_LSTM	Hybrid_LSTM
Accuracy	0.9498	0.9595	0.9371	0.9431	0.9639	0.9787	0.9908
Variance	0.0297	0.0292	0.12	0.0564	0.0276	0.0266	0.0051
Time (s)	0.001	0.001	0.0011	0.0024	0.0087	0.0018	0.0063

**Table 5:** Performance of normal vs. nonseizure case (AB vs. CD) with 10-fold cross-validation.

Methods	K1	K2	K3	K4	K5	K6	K7	K8	K9	K10	Mean	Variance
EEG	0.9806	0.9667	0.9667	0.9722	0.9667	0.9806	0.9861	0.9556	0.9861	0.9417	0.9703	0.0141
DWT	0.9694	0.9750	0.9639	0.9722	0.9528	0.9806	0.9833	0.9167	0.9306	0.9472	0.9592	0.0221
FFT	0.8556	0.8556	0.8444	0.8361	0.7222	0.8167	0.8583	0.8694	0.8444	0.6	0.8103	0.0849
STFT	0.9917	0.9778	0.9861	0.9611	0.9417	0.9833	0.9917	0.9750	0.95	0.9417	0.97	0.0198
Hybrid	0.9917	0.9778	0.9833	0.9778	0.9722	0.9889	0.9889	0.9556	0.9833	0.9694	0.9789	0.011

## Data Availability

The adopted EEG dataset is acquired online, which is published by Andrzejak et al. [27]. Other data used to support the findings of this study are available from the author upon request (jianxiangwu991230@126.com).
